RETRACTED

# Application of BIM Technology in Prefabricated Buildings Based on Virtual Reality

**DOI:** 10.1155/2022/9756255

**Published:** 2022-10-03

**Authors:** Wei Zheng, Yong Ye, Hongbing Zang

**Affiliations:** Construction Management and Real Estate Department, Tongji University, Shanghai 200092, China

## Abstract

Prefabricated construction is an emerging technology in the construction industry, which can effectively meet the construction scale requirements of construction projects. It can also shorten the construction time and reduce unnecessary consumption of construction resources. The introduction of BIM + VR technology into the prefabricated construction industry will improve and improve the construction of the relevant construction industry chain, architectural visualization design, architectural virtualization construction, project cost management, and production operations. In particular, the application of BIM + VR technology to the construction of prefabricated buildings can further refine the entire construction process and improve the overall quality of the project. The application advantages of these two technologies are analyzed, and the practical application of advanced technologies in building construction is discussed for reference.

## 1. Introduction

At this stage, my country's urbanization construction process is continuing to deepen. Relevant research shows that about 40 billion square meters of buildings have been built in my country, of which 95% are high-energy-consuming buildings. The number of buildings of this type is also increasing with the deepening of construction [1, 2]. Such a high proportion of energy-consuming building forms not only create a significant energy burden. It also directly restricts the growth of the national economy, has an impact on the ecological environment, and reduces the quality of life in harmony between man and nature.

Based on this, the green concept is increasingly emphasized in construction projects, and the energy saving and environmental protection of buildings are emphasized. However, the traditional construction method of construction industry no longer meets the needs of modern development of the construction industry. As a typical representative of green buildings, prefabricated buildings refer to building products that are prefabricated in factories, assembled and installed at the construction site, and finally connected by mortar anchors or post-cast concrete. Compared with traditional cast-in-place construction operations, the construction form of prefabricated buildings has significant advantages such as shortened construction period, reduced on-site labor, improved construction quality, and more convenient information management. Promoting the development of the prefabricated construction industry has become an important path for the transformation and upgrading of the construction industry in the next step.

RETRACTED

With the continuous development of computer and information technology, building information model software technology is becoming more and more mature. As a hot technology and research hotspot in the field of construction engineering in recent years, BIM (building information modeling) is based on three-dimensional digital technology. It integrates all kinds of related information data in construction projects to build models, which is an intuitive display and detailed expression of engineering information [3, 4]. At the technical level, it has seven characteristics, including simulation, optimization, visualization, cost controllability, coordination, plotting, and cost accuracy. VR (virtual reality) was proposed in the early 1980s, which is a new form of human-computer interaction created by the combination of computer and advanced sensing technology. VR technology is one of the most influential technologies in various fields at present and has wide application prospects in various fields.

It can be seen from the above that prefabricated buildings have higher requirements for construction technology, technical parameters, material composition, and engineering personnel. Therefore, through the application of new technologies, focusing on the improvement of enterprise construction capabilities, the cultivation of relevant professionals is particularly important in the entire industrialization system of the construction industry [5]. In response to the above problems, BIM + VR technology should be introduced into the prefabricated construction industry. It will improve and improve the construction of related construction industry chain, architectural visualization design, construction virtualization construction, project cost management, and production operation.

## 2. Overview of Prefabricated Buildings

### 2.1. Concept of Prefabricated Buildings

The Western Industrial Revolution has greatly improved the production efficiency of manufacturing industries such as shipbuilding and automobiles. In the 1920s, the new building movement of modular production of components and on-site construction and assembly was the early prototype of prefabricated buildings. After World War II, a large number of buildings in Western countries were destroyed, and the national housing problem needed to be solved urgently. Prefabricated buildings are highly praised by countries because of their high work efficiency. In the 1960s, there was another wave of prefabricated buildings that focused on quality and efficiency in Western countries.

RETRACTED

As a developing country, my country's prefabricated buildings started late compared with the country. In the 1950s, the Ministry of Construction issued the Outline for the Development of Industrialized Buildings, which clearly put forward the concept of industrialized buildings. That is, the construction industry should gradually transition from the traditional labor-intensive manual production mode to the mechanized large-scale production mode. It adopts advanced technology and mechanical equipment to develop the production of building components, products, and equipment on the basis of meeting building specification. Subsequently, the State Council issued the “Decision on Strengthening and Developing the Construction Industry.” It is proposed that to fundamentally change the construction industry in our country, it is necessary to actively implement the mechanization and modularization of construction and gradually realize the transformation from traditional buildings to industrialized buildings [6]. Since then, the prefabricated building industry has gradually entered the public's field of vision in my country and has attracted extensive research and attention from scholars.

In summary, prefabricated buildings use factory-made prefabricated building components, which are transported and hoisted on-site to form a complete building structure. This greatly accelerated the construction progress, mainly including fabricated concrete structures, steel structures, and wood structures.

### 2.2. Characteristics of Prefabricated Buildings

Due to the different focuses of different scholars and experts, there are also different views on the early understanding of prefabricated buildings. After a lot of theoretical and practical research, scholars generally believe that prefabricated buildings have the following “four modernizations” characteristics.

#### 2.2.1. Standardization of Architectural Design

Standardization of architectural design is the basis and premise for the realization of prefabricated construction. Compared with cast-in-place structures, a distinctive feature of prefabricated buildings is modular design and production. This requires the components to be as consistent as possible in terms of type, size, and material [7]. This can not only greatly shorten the design cycle but also reduce the design cost and construction cost. It can also facilitate the production, transportation, and installation of the components and greatly ensure the construction quality of the components.

#### 2.2.2. Factory Production of Components

The core feature of prefabricated construction is factory production. As the basic parts and components of buildings, components are extremely important in their production and production processes. It is based on standardized design, and the factory realizes unified production and manufacturing. It not only has the characteristics of batch and high efficiency but also greatly improves the production quality of components compared with the cast-in-place structure.

RETRACTED

#### 2.2.3. Construction Assembly

Construction assembly refers to the process of splicing and assembling factory-produced prefabricated components at the construction site. Compared with traditional cast-in-place operations, prefabricated buildings are less affected by climate and environment. The notable features of construction assembly are the high degree of mechanization, the small on-site workload, the decrease in the number of operators, and the significant improvement in construction efficiency. It not only reduces energy consumption and construction waste emissions but also greatly reduces disturbance to the surrounding environment.

#### 2.2.4. Management Informatization

In the whole life cycle of a construction project, compared with the industrial production and installation of buildings, the operation management of buildings is also very important. Advanced informatization means (Internet, BIM, etc.) should be used for the operation and management of buildings. The application of information technology is not only an important guarantee for realizing the industrialization of construction. At the same time, it is also an important tool to realize the whole-process monitoring and information management of design, construction, and operator. This can greatly improve the engineering quality and construction efficiency of prefabricated buildings.

### 2.3. Difference between Prefabricated Construction and Traditional Construction

Compared with the traditional construction method of cast-in-place structures, prefabricated buildings have unique advantages in the design stage, construction process, and management system. While ensuring quality, it can not only increase productivity and improve construction environment but also significantly optimize project quality and improve project efficiency. The comparison between traditional construction and prefabricated construction is shown in Table 1.

### 2.4. Development Status of Prefabricated Buildings

Prefabricated buildings appeared earlier in developed countries such as Europe and the United States. Since the 1970s, the United States began to promote the construction of building accessories and mechanized production. As early as the 1950s, my country proposed to promote the development of related industries, but due to limited construction capacity and weak economic foundation, the development of the industry was greatly hindered. It is required to strive to make prefabricated buildings account for 30% of the new construction area nationwide in the next 10 years or so, and its development prospects are huge.

RETRACTED

In recent years, major cities in China have actively issued policies and guidance documents for the promotion of the prefabricated construction industry. It is also required to use prefabricated building construction to complete the construction of residential security housing. The sustainable development of prefabricated buildings in China is inseparable from policy support and market orientation [8]. Many real estate companies are also gradually participating in the industrial exploration of prefabricated buildings. It can be seen that the development conditions of domestic prefabricated buildings are gradually improving and strengthening.

However, there are two major problems in the development of the domestic prefabricated construction industry. ① Professional talents are in short supply. At present, the talent training and management system of the domestic construction industry has not yet adapted to the development needs of prefabricated buildings. Major secondary schools lack relevant professional settings and lack channels for training skilled workers. ② It is difficult to promote technology. Industry technical barriers lead to high barriers to entry, directly hindering the transformation, progress, and interaction of enterprises. As far as the current situation is concerned, prefabricated buildings only account for 5% of the new construction area. The lack of scale effect makes the cost higher than the traditional method, and the technical threshold is high, making it difficult to expand the scale.

In the existing teaching and construction training for prefabricated buildings, there are problems of high cost, high difficulty, poor repeatability, and operability. Teachers have problems that the guidance is not intuitive enough and the demonstration is not clear. However, the teaching object can also feel more abstract in the process of accepting the learning. Combined with the factors of insufficient operability, it is more difficult to accept the ability.

## 3. BIM and VR Technology

### 3.1. BIM Technology

#### 3.1.1. Definition of BIM

BIM is actually short for building information modeling. In the construction industry, the process of using a modern digital model management system to optimize the overall control of a construction project is called BIM. It applies to all phases of construction project operation. In addition, the model in the BIM model refers to the method and utilization, and the information is divided into two types. One is information of nongeometric properties, and the other is information of geometric properties.

RETRACTED

In fact, BIM is the International Building Information Modeling Standard in the standardized translation of the United States. Its standardized definition is to use a digital information model to record the specific content and related information of the project, so as to provide a reliable basis for the opening and progress of the construction project [9]. BIM is not only for a complete project but also can be controlled by BIM for the project under construction, and the information corresponding to the project can be adjusted according to the changes.

Nowadays, the level of social science and technology is constantly developing in various industries. As a new concept and new technology to promote the development and innovation of the construction industry, BIM has attracted the attention of a large number of scholars and industry-related personnel at home and abroad. The first revolutionary innovation in architectural engineering actually refers to the transition from drawing boards to CAD (computer-aided design). The application of BIM technology from two-dimensional to multidimensional will become the second revolution of the entire construction industry.

#### 3.1.2. Characteristics of BIM Technology Applied to Prefabricated Buildings

Prefabricated buildings are characterized by standardized components and information management. However, the advantages of BIM technology application can perfectly meet the needs of the development of prefabricated buildings. To realize the development of building industrialization, the integration of prefabricated buildings and BIM technology is the inevitable result of the integration of building industrialization and building informatization.

Today, with people's increasing requirements for construction, the traditional construction model has been unable to adapt to the rapid development of today's construction industry, and the rise of prefabricated buildings has become inevitable. Among them, the intervention of BIM technology also plays an indispensable and important role in the development of prefabricated buildings. BIM technology plays a role in information transmission and interaction in the design, construction, deepening, and other stages of prefabricated buildings. It improves the efficiency and provides a new management method through its own unique information clustering function in many aspects such as management, operation, and collaboration. Prefabricated buildings are different from traditional building models. Efficient information transmission, professional collaboration, and refined management have promoted the continuous innovation of prefabricated building technology. At the same time, it has also continuously promoted the rapid development of China's construction industry.

RETRACTED

In the whole life cycle of building construction, prefabricated structures have problems such as complicated management work and easy distortion of construction data. BIM technology can realize information management and efficient interaction at all stages. It is not only conducive to the realization of green construction, safe construction, and civilized construction of prefabricated buildings during the construction process but also to achieve precise and efficient management, which can greatly reduce the demand for construction resources. At the same time, it is also conducive to environmental protection, effectively controlling costs, and promoting the sustainable development of prefabricated buildings.

Over the years, the application of BIM technology in actual engineering projects has continued to develop with the development of the construction industry. From the initial construction of 3D models, to the later platform-based collaboration, green building simulation, and building in-depth design, all aspects are constantly innovating. It promotes the Chinese construction industry to get rid of the inherent old thinking mode, which is beneficial to the healthy development of the construction industry.

BIM technology is used in many fields in prefabricated buildings. It is involved in the establishment of standardized family libraries, component production, preassembly inspection, construction process simulation, material management, collision detection, information management, equipment troubleshooting, and emergency plan formulation. The specific points are as follows:

1. The design process can be accelerated, the prefabricated components can be reused after the design is completed, and the design can also be quickly assembled and drawn.
2. BIM technology can carry out refined three-dimensional modeling, assisting the high-precision prefabrication of standard components in the factory. In addition, the use of BIM technology for on-site construction simulation can ensure the reasonable assembly of prefabricated components and avoid delays such as rework.
3. It can be better connected to guide prefabrication and can be connected to automated prefabrication equipment. Prefabrication automation can be combined with 3D scanning and other means to compare prefabrication and design errors before leaving the factory and can also guide the construction process through simulated construction.

RETRACTED

#### 3.1.3. BIM Technology Combines the Advantages of Prefabricated Buildings

1. In the whole process of design and construction of prefabricated construction projects, the intervention of BIM technology can make management more precise and efficient than before. It can not only meet the requirements of national policies in terms of construction quality and safety but also have a positive impact on resource conservation and environmental protection.
2. With the vigorous development of prefabricated buildings, the transformation and innovation of construction technology have become an indispensable step in the development of the construction industry. Based on the development of BIM technology, not only can new and old technologies in our country be constantly updated and new but also can continuously promote the industrialization of my country's construction industry.
3. The comprehensive management of green construction runs through the whole life cycle of the prefabricated building project, and the prefabricated building construction requires that the environmental pollution be minimized. The application of BIM technology to green construction can help optimize construction management, reduce environmental impact, and save resources.
4. BIM technology can provide a strong guarantee for the growth of prefabricated buildings.

### 3.2. VR Technology

Virtual reality, as its name implies, simulates the existing environment and things and creates a new virtual reality space through a computer. However, as we all know, the real environment is so complex that it not only exists in the plane visual effect, but even achieves a three-dimensional dynamic effect, and has a unique existence in many aspects such as smell and hearing. Therefore, virtual reality technology is a combination of various disciplines and technologies, including human-machine interface technology, sensing technology, simulation technology, and network sensing technology [10]. The ideal state of virtual reality is like creating another real scene. The creation of the scene actually needs to integrate a variety of information, and the simulation of the environment is actually realized by the generation of three-dimensional animation by the computer. VR is a multi-sensing effect created by sensing devices, that is, a three-dimensional interactive system. Due to the joint participation of a variety of high-end technologies, virtual reality technology is also a high-end project that is at the forefront of science.

Of course, VR technology cannot be achieved overnight. In fact, it has gone through four different stages. The first stage was before 1963, and it was called acoustic dynamic simulation and included the idea of virtual reality. The second stage (1963–1972) was the germination period of virtual reality. VR formed related concepts and related theories in the third stage, that is, from 1973 to 1989. The virtual reality theory was further supplemented and applied in the fourth stage (1990–2004).

RETRACTED

#### 3.2.1. Multisensitivity

Multisensibility not only refers to the visual perception brought by ordinary computer images but also involves more perceptual content, such as touch, smell, and hearing, and even includes taste perception and motion perception. An ideal virtual reality should have all the perceptual capabilities of a human.

#### 3.2.2. Sense of Existence

The sense of presence is that the user feels that he is the protagonist in the simulation environment. The ideal simulation environment should be a virtual environment where it is difficult for the user to distinguish the true from the false.

#### 3.2.3. Interactivity

Interactivity mainly refers to the interaction between the user and the simulated environment, that is, what the user can do in the face of the virtual environment and what can the environment give back to the user.

#### 3.2.4. Autonomy

Autonomy refers to the degree to which objects in the virtual environment function according to the laws of physical motion in the real world.

### 3.3. Hybrid Technology of BIM + VR

The hybrid technology of BIM + VR brings users a wonderful experience by introducing real scene information into the simulated VR scene. Establishing information exchange between users and real scenes and virtual scenes is a further development of VR technology. The hybrid technology of BIM + VR refers to the creation of new visual effects by merging the virtual world with the real world. Moreover, in such a new visual environment, digital objects and physical objects exist at the same time, and there are exchange and interaction of information between them. The hybrid technology of BIM + VR has the following three characteristics:

1. Combining virtual scenes with reality
2. Applying 3D stereoscopic effects to virtual scenes
3. Real-time operation

The hybrid technology of BIM + VR is more demanding than VR and AR technology. It pursues the interaction between virtual and real scenes, and as VR only needs to realize the construction of virtual scenes, AR just superimposes the virtual scene and the real scene. Therefore, the key of mixed reality technology lies in the information interaction with reality, and it is necessary to obtain the information of the real scene in time and make a response. It is not only “mixed reality” but also “the father of intelligent hardware,” the concept of “intermediate reality” proposed by University of Toronto Professor Steve Mann.

RETRACTED

In the 1970s and 1980s, Steve Mann designed wearable smart hardware to enhance its own visual effects and see the surrounding environment no matter what the scene is, which is considered an initial exploration of MR technology.

VR is a pure virtual digital image, and MR is a digital reality plus virtual digital image. In theory, MR and AR are more similar, and they are both semi-real and semi-virtual images. However, traditional AR technology uses prism optics to refract the real image, which affects the clarity of the image, and the perspective effect is not as great as that of virtual reality [11].

MR technology combines the advantages of VR and AR, and it can better reflect AR technology. Steve Mann once said in the theory that the AR technology in the intelligent system of today's society will eventually go to MR. Reality hybrid technology allows people to see the real world that is invisible to the naked eye through only one camera, which is what differentiates it from AR.

## 4. Application of BIM + VR Technology in Prefabricated Buildings

### 4.1. Implementation of BIM + VR Technology in Prefabricated Buildings

BIM and VR technology is applied to prefabricated buildings to virtualize and reproduce building construction. It is converted into a specific digital animation using related technology, and the corresponding architectural parameters are obtained through the related view method. In this process, the use of VR technology can realize the simulation and reproduction of each link in the construction process of the prefabricated building [12]. On this basis, the reproduction and simulation of the construction process are realized, and the best construction plan and technical parameters are obtained through a comprehensive investigation of the relevant factors, which lays the foundation for achieving a good construction effect. In addition, using BIM and VR technology can also realize one-to-one component query, organically reproduce the construction process of prefabricated buildings, and bring a vivid and concrete reality reproduction system to the staff. In the specific production and construction process, this system can be used for specific construction training and overall construction. It is helpful to realize the overall optimization and coordination of the construction industry and realize the effective control of the whole construction process.

With the continuous innovation of new technologies, the traditional construction industry has undergone subversive changes. As an important achievement in promoting the development and innovation of the construction industry, the hybrid application of BIM + VR technology has a huge impact on the progress and transformation of the construction industry. Due to the technical reasons of workers, the quality level of the construction site samples built with traditional technology is usually uneven, and the site demand is large, the material consumption is large, the waste is obvious, and it is difficult to recycle and reuse. However, by introducing the building model constructed by BIM + VR technology, observers can not only enter the virtual environment but also observe and learn about the typical operation process, detailed nodes, and construction technology. It can also improve the design quality with reasonable planning in the site layout and achieve the predetermined goal of environmental protection and efficiency.

RETRACTED

In addition, the construction materials required for the building are simulated in the virtual environment, and the experience will be more intuitive through modules such as material changes, lighting difference simulation, and internal living facility layout. Compared with traditional technologies, the application of new technologies is more in line with the requirements of green buildings [13]. That is, it can be recycled, which can directly and effectively avoid the waste of materials, human resources, and the standardization of construction models caused by differences in the technical level of workers.

At the same time, the hybrid application of BIM + VR technology will solve the current biggest pain point in the construction industry, that is, “what you see is not what you get” and “engineering control is difficult,” and the control difficulty lies in the overall planning, integration of resources, abstract association, and platform construction. Through the systematic design of the BIM platform, while strengthening the project management ability, the architectural design process will be further informatized and three-dimensionalized. The introduction of VR, on the basis of BIM 3D model, will enhance concreteness and visibility. Building a virtual display can provide users with house-type design and visual intuitive display. The BIM + VR model is expected to provide solutions to industry pain points, promote the emergence of new business forms, and greatly enhance the application effect and depth of BIM technology.

### 4.2. Application Characteristics of BIM + VR Technology

#### 4.2.1. Simulation

With the continuous expansion of the scale of construction projects, it is difficult to realize the expected analysis of work requirements only with the help of BIM building model technology. To further strengthen the work effect, it is necessary to integrate virtual reality technology. According to various building data information, the building construction process is realized. For example, the building model system platform is used to input various building materials and construction technology information into the model and accurately mark the sequence process of each construction. In this way, the system can simulate the construction scene according to the data information. The system platform can not only combine with 3D building model technology to strengthen the visualization of simulation results but also has good information interaction function. For example, in the simulation stage, technicians can replace related operations, see the application effect after the adjustment of the construction plan, visualize the matching plan of the construction technology, and present it in the form of a three-dimensional model. If the planned scheme is feasible, the subsequent construction content can be adjusted in time, and the design scheme can be continuously optimized during the construction process.

RETRACTED

#### 4.2.2. Application Characteristics

VR technology has features such as rendering advantages, particle effects, new material pipelines, and blueprint systems in applications. The main advantages are as follows. ① Visualization technology has good image display effect and can accurately convert preset values. The combination of displacement technology and mosaic technology makes the simulation effect of specific objects more vivid and clear. ② The particle effect editor is mainly used in various reproduction and simulation and reorganizes the detailed data according to the dynamic characteristics of particles. It can achieve effective control of particle parameters, including color, size, and density, and can more comprehensively reflect the actual situation of the building [14]. ③ The new material pipeline provides technicians with a new management and control method, which makes the virtual simulation scene more open, and the material characteristics can be adjusted according to actual needs. Thereby, the best matching scheme is obtained, so that the relevant technical parameters can meet the construction quality requirements. ④ The blueprint system can help technicians to expand their ideas and further broaden their horizons. Various adjustment methods are reflected in specific visualization models to accurately determine the practical application effects of various design ideas.

#### 4.2.3. Achievement Display

In practical applications, both BIM technology and VR technology can be connected with the operation platform for data connection, and the data information is effective and universal. For example, the blueprint system is used to analyze the construction effect of prefabricated buildings, and technicians can reproduce the situation according to the model. Data information is integrated and optimized to make the overall architectural model more vivid and realistic. For construction materials, the subsequent material surplus can be calculated according to the loss of each construction stage. Starting from the overall level of the project, the loss of various construction resources is accurately coordinated. Technicians can compare different plans horizontally from various aspects to find out the most cost-effective architectural plan. In addition, in the combined system of BIM technology and VR technology, the platform can also strictly control construction personnel and specific processes. For example, if the construction personnel wear the positioning device, they can realize the position control of the whole construction site and greatly improve the construction safety and quality.

RETRACTED

#### 4.2.4. Process Simulation

The process simulation of prefabricated engineering should first use BIM building model technology to integrate and reproduce the data information in the construction stage and then simulate the whole process of construction. This type of technology is mainly used in the connection and cross-operation of each construction stage, and the technicians can correspond to the components according to the construction. The construction process and display system are inquired, and the materials required for each construction technology are accurately grasped [15]. The construction process is fully controlled, and it is turned into a concrete visualization system. At the same time, the process simulation should be carried out in strict accordance with the data parameters in the construction plan. Only in this way can the deficiencies in the design scheme be accurately reflected.

### 4.3. Application of BIM + VR Technology in Prefabricated Buildings

#### 4.3.1. Split Design of the Whole Process of Prefabricated Construction

The application of BIM technology and VR technology in the construction of prefabricated buildings can adopt the whole-process split design mode, that is, to carry out refined management and control of the entire construction process, focusing on the analysis of spatial environmental information. At the same time, it can accurately determine the application effect of various building components, reasonably reduce the types of exterior wall components and floor components, and improve construction quality and efficiency. The split design process is shown in Figure 1. First, the CAD graphic information is identified and the relevant data are extracted into the BIM building model. The data parameters of the BIM building model are successfully read to realize the construction process and component conditions. In the detailed analysis of the specific construction stage, the combination scheme of the prefabricated components can be split to form an accurate and clear split diagram. Technicians can adjust and replace various components to optimize the construction material scheme.

RETRACTED

#### 4.3.2. Application Process Based on BIM and VR Technology

The BIM building model technology is applied to realize the splitting of the prefabricated structures in each construction stage. Beams, slabs, columns, walls, and other components can be reorganized to form a new CAD graphic. For example, to split prefabricated beams and slabs, it is necessary to establish BIM model families of various beam-column joints according to the BIM model of the prefabricated building. According to the connection between different nodes, the parameter situation is displayed in the node family. The building model is split through the optimization algorithm to accurately reflect the application coefficient of the shear wall structure. In addition, on the one hand, starting from the application quality, the overall quality of the prefabricated building can be calculated by replacing various prefabricated components [16]. On the other hand, we can start from the loss of construction resources and cost expenditure and choose the scheme with the least application of construction resources, to improve the profit and efficiency of construction enterprises.

#### 4.3.3. Strengthen the Exchange of Construction Information

The application of BIM technology and VR technology to the construction of prefabricated buildings can also strengthen the exchange of construction information. For example, in the early scheme design, adjustment and optimization, and construction deployment, more manpower and material resources need to be invested, and the actual implementation effect is poor, and it needs to be adjusted and optimized repeatedly. The VR virtual simulation technology can accurately visualize various data information. The construction content is clearly divided into specific positions and personnel and is linked to the construction responsibility management system, so that the refined management work has a clear direction. On this basis, real-time communication is carried out, and the relevant personnel are urged to inspect the construction plan and feedback their opinions to the technical department in a timely manner [17]. Various construction quality problems can be dealt with in advance, greatly reducing hidden dangers in the construction process.

RETRACTED

In the construction process of prefabricated construction projects, it takes a lot of manpower and material resources in the early drawing review, design optimization, visa construction, etc. To save resources, VR technology can be used for effective work. The specific content of specific links in the construction process is converted into corresponding staff objects, and specific work tasks are assigned to them [18]. On this basis, real-time communication is carried out, and relevant personnel are urged to accurately observe and inspect the construction plan, and feedback on their opinions is given timely. Finally, an overall construction plan is obtained, which lays the foundation for achieving a good overall construction effect and laying a foundation for improving the construction quality. In this process, the overall construction plan will be effectively promoted, laying a foundation for further improving the construction effect and progress.

#### 4.3.4. Realize Refined Cost Control

For contemporary construction enterprises, to ensure a good competitive advantage in the industry market, they must optimize and innovate construction technology and materials and continuously improve the quality of construction projects. However, various advanced technologies and new materials will involve more cost expenditure, and each construction stage faces a large amount of construction resource loss. Therefore, using BIM technology and VR technology, it is necessary to carry out refined management and control of construction costs. The whole process in the early stage of construction is simulated, and the material quantity and loss degree required for each construction link are accurately calculated, which can provide accurate data support for construction site management. In addition, in the construction of large-scale construction projects, the management decision-making of each construction link should also rely on BIM architectural model technology. By calculating the construction volume, rationally deploying construction personnel and work content, and eliminating redundant construction teams, it has good application value and practical value to realize the optimal allocation of human resources.

Using VR technology, the specific construction links of prefabricated building construction can be reproduced and simulated. According to the virtual effect, a scientific and effective construction plan can be obtained, and the relevant construction links can be controlled as a whole, which can effectively save resources and avoid a lot of waste of resource costs in the construction process. In this process, VR technology can accurately reproduce the specific links of prefabricated building construction. This process can provide necessary help to explore the best construction scheme and also provide necessary help to study how to effectively save resources in the construction process. The staff can simulate the building construction plan, specific materials, construction process, etc., on-site. On this basis, the advantages and disadvantages of specific construction schemes and cost control can be analyzed. This process helps the staff to grasp the specific construction process, cost control effect, overall construction cost, and economic benefit of each scheme. By comparing the advantages and disadvantages of specific schemes, the best construction scheme is obtained, thereby greatly reducing the waste of resources in the practical construction process and realizing the optimal allocation of human resources. It promotes each link of building construction to achieve the best economic and social benefits in the practical process and has good application value and practical value.

RETRACTED

#### 4.3.5. Analyze the Execution Effect of the Construction Plan

Finally, it is necessary to ensure the implementation of the construction plan. In the virtual reproduction of VR, the content of the construction plan is gradually displayed. For example, decision-makers and technicians can enter the building model, observe the building as a whole from any perspective, and observe the building results in detail from the application of materials, lighting conditions, and real locations. Using BIM technology to establish engineering models, construction personnel can also intuitively feel the construction site environment and find out possible problems in the construction process. This can not only improve the construction quality and efficiency but also strengthen the construction personnel's awareness of the safety and quality of the project. In the actual operation, it can be implemented according to the pre-deployed plan and has an accurate grasp of construction technology, design principles, and force analysis. Therefore, construction companies should also strengthen the technical level training of construction personnel, so that they can more proficiently use BIM technology and VR technology to improve the overall quality of the construction team.

#### 4.3.6. Prefabricated Construction Training and Management

VR technology can turn architectural plans on two-dimensional drawings into models with a more spatial sense. Decision-makers can enter the mock-up at will, experience and observe the works from any perspective, from materials, dimensions to lighting, and experience the location scene and spatial dimensions in real terms. The engineering model established by BIM technology is combined with VR experience equipment to realize dynamic roaming, and the BIM model disclosure has a more realistic experience. The construction personnel can feel the construction site more intuitively, help the construction personnel understand the construction plan and construction technology, and improve the construction quality [19]. Today's buildings are becoming more and more peculiar in shape, and their internal design structures are becoming more and more complex. Through VR virtual experience technology to understand the corresponding methods in architectural design and construction, you can have a comprehensive understanding of the design principles, construction technology, force analysis, and pipelines of such buildings. In the practice process, the staff can effectively online the entire construction process of the prefabricated building and use virtual reality technology to achieve accurate simulation of various construction details. On this basis, the construction personnel are organized to observe and reproduce the workflow, work details, work practice techniques, and places that need attention. The staff are helped to accurately grasp the details of the overall construction process through this process, and the foundation is laid for subsequent related construction and construction training work, bringing more vivid and accurate practical training effects to the staff. It can promote the construction team to grasp the overall construction project and play a role in promoting the realization of a good overall construction effect.

RETRACTED

BIM technology has changed the traditional construction method in the construction method, and the birth of VR virtual reality technology has brought people different perceptions and interactions. The combination of the two is bound to enhance the technical level of each other. Model house roaming and virtual disclosure are just the beginning of the integration of VR and BIM. In the future, BIM and VR system platforms can be used to build virtual cities. It provides possibilities for urban creation and promotes the development and change in large cities.

## 5. Conclusion

With the help of BIM technology and VR technology to innovate the traditional construction mode, it can strengthen the fit between the construction plan and the actual implementation and accurately control the resource consumption in each construction stage. The combination of the two technologies will continue to expand to a deeper level, which is conducive to the smooth development of large-scale construction projects. This study studies the application of prefabricated building technology under the background of BIM technology and VR technology. Firstly, the concept and characteristics of BIM technology and VR technology are expounded, and then, the application of the two technologies is analyzed. Finally, the practical application results of advanced construction technology in current construction projects are presented. Based on the application process of BIM technology and VR technology, the exchange of construction information is strengthened, refined cost control is realized, and the effect of construction plan execution is analyzed. It can provide assistance for the good development of construction enterprises.

RETRACTED

## Figures and Tables

**Figure 1:** Split design process of construction engineering.

**Table 1:** Comparison of traditional construction and assembled construction.

Construction methods	Stage	Main contents
Traditional construction method	Design	Only starting from the architectural design structure, without considering the construction method, construction technology, etc.
	Construction	Workers put production factors on-site by themselves, mainly manual work, and the production efficiency is low
	Management and benefits	The design-production-construction links are separated, the industrial chain is scattered, management is difficult, and enterprise efficiency is low

Prefabricated building construction method	Design	The design is matched with standardization and systematic integration technology, pays attention to the coordination and cooperation of the industrial chain, and considers the modules and standards of the components, the integration technology and parameters of the building system, etc.
	Production	The proportion of components and production factors is carried out according to the design requirements, and the production is unified in the factory, and the production efficiency is high
	Construction assembly	On-site assembly of components and building systems, integration of construction and design, and factory production
	Management and benefits	The whole process of the design-production-construction link is intensive and information-based, which creates higher corporate benefits

## Data Availability

The dataset can be obtained from the corresponding author upon request.
